RETRACTED

# Different azithromycin protocols for management of preterm prelabour rupture of membranes: a randomized clinical trial

**DOI:** 10.1186/s12884-022-05189-7

**Published:** 2022-11-23

**Authors:** Laila Ezzat Abdelfattah, Rehab Abdelhamid Aboshama, Amr S. Abdelbadie, Mohamed H. Abulhasan, Mohamed A. Anan, Ibraheem I Abdelaal

**Affiliations:** 1 Associate professor of Obstetrics and Gynecology, Department of Obstetrics and Gynecology, Faculty of Medicine, Fayoum University, Fayoum, Egypt; 2 Lecturer of Obstetrics and Gynecology, Department of Obstetrics and Gynecology, Faculty of Medicine, Fayoum University, Fayoum, Egypt; 3 Lecturer of Obstetrics and Gynecology, Department of Obstetrics and Gynecology, Faculty of Medicine, Aswan University, Aswan, Egypt; 4 Resident of Obstetrics and Gynecology, Department of Obstetrics and Gynecology, Faculty of Medicine, Aswan University, Aswan, Egypt; 5 Lecturer of Obstetrics and Gynecology, Department of Obstetrics and Gynecology, Faculty of Medicine, Assiut University, Assiut, Egypt

**Keywords:** Azithromycin, Latency period, Chorioamnionitis, Preterm Pre-labor Rupture of Membranes, Neonatal outcomes

## Abstract

**Background:**

Preterm prelabor rupture of membranes is associated with polymicrobial infection; hence broad-spectrum antibiotics are recommended**.** Nowadays, Azithromycin is used instead of Erythromycin due to erythromycin shortages, its ease of administration, decreased cost, and better side effect profile. This study aimed to evaluate the efficacy of different azithromycin protocols for the conservative management of preterm prelabor rupture of membranes.

**Methods:**

It was a single-blinded randomized clinical trial including pregnant women at 24–36^+6^ weeks with viable singleton pregnancies and confirmed preterm prelabor rupture of membranes from January 01, 2020, to June 01, 2021. The participants were randomized into two groups: Group I was made of women who received Azithromycin 1000 mg PO once, and Group II of women who received Azithromycin 500 mg PO once, followed by Azithromycin 250 mg PO daily for four days. The primary study outcome was the length of the latency period from the diagnosis of preterm prelabor rupture of membranes to delivery (days).

**Results:**

The latency period in group I was significantly higher than that in Group II (5.80 ± 5.44 days vs. 2.88 ± 2.37; respectively, *p* = 0.0001). The mean gestational age at the time of delivery was significantly higher in Group I (*p* = 0.0001). However, postpartum endometritis and respiratory distress syndrome (RDS) rates were significantly higher in Group II (*p* = 0.003 and *p* = 0.0001, respectively).

**Conclusion:**

The higher dose of Azithromycin was associated with better maternal and neonatal outcomes.

RETRACTED

**Trial registration:**

Clinical trial identification number: Clinical trial.gov: NCT04202380 (17/ 12/ 2019).

Date of registration: 1/1 /2020.

Date of initial participant enrollment30 /1/2020.

URL of the registration site: https://www.clinicaltrials.gov/ct2/show/NCT04202380

## Background

*Preterm premature rupture* of membranes (PPROM) is defined as the spontaneous rupture of fetal membranes before 37 completed weeks of gestation. PPROM complicates approximately 3% of pregnancies and is associated with 30%–40% of preterm births [1, 2]. Rupture of membranes **(**ROM) is diagnosed via the patient's history, followed by a sterile speculum examination. If no amniotic fluid is observed, insulin-like growth factor-binding protein-1 (IGFBP-1) or placental alpha microglobulin-1 (PAMG-1) tests are carried out to confirm the diagnosis (3**).**

PPROM is associated with an ascending infection that leads to chorioamnionitis and fetal and neonatal infections [4]. Microorganisms are present in approximately 30% of PPROM cases [5]. The frequency of infection increases over the latency period; so, when a patient with PPROM goes into active labor, microorganisms are detected in 75% of cases [6].

The management between 24 and 37 weeks includes hospital admission, fetal monitoring, assessment of infection, and courses of corticosteroids and antibiotics to prolong the latency period between PPROM and delivery [3]. The American College of Obstetricians and Gynecologists (ACOG) recommends broad-spectrum antibiotics in cases of PPROM because the infection is polymicrobial**.** Many antibiotic regimens have been found to prolong the latency period [5].

Intravenous Erythromycin and ampicillin for two days, followed by oral Erythromycin and amoxicillin for five days, is the most common regimen used in PPROM that the ACOG supports. This regimen was associated with prolonged latency to delivery and a decrease in the incidence of chorioamnionitis and fetal/neonatal complications [6]. Nowadays, Azithromycin is used instead of Erythromycin due to its ease of administration, decreased cost, better side effect profile, and erythromycin shortages [7, 8]. There is a need to evaluate the effect of different azithromycin protocols on the latency period in women with premature rupture of membranes. The current study hypothesized that a single dose regimen of Azithromycin would be associated with prolonged latency period than the multiple dose regimen.

## Methods

The study was a single-center, a single-blinded, randomized, parallel clinical trial carried out from January 01, 2020, to June 01, 2021, at Aswan University Hospital. We included women according to the following inclusion and exclusion criteria. The inclusion criteria were a) viable singleton pregnancies, b) gestational ages of 24–36 + 6 weeks, and c) confirmed PPROM diagnosed via maternal history and sterile speculum examination demonstrating liquor. The exclusion criteria were a) women presenting in labor, b) fetal death, c) congenital fetal anomalies, d) patients refusing to participate in the study, e) unconfirmed gestational ages, f) macrolide allergy, g) women who received macrolide therapy within a week before recruitment, h) and contraindications to the expectant management of PPROM at the time of diagnosis such as concurrent preterm labor, placental abruption, chorioamnionitis diagnosed by the presence of fever ≥ 37.8◦c and at least 2 out of the following; total leukocytic count > 15,000, maternal tachycardia > 100 beats per minute, fetal tachycardia > 160 beats, uterine tenderness, and offensive vaginal discharge [9], or non-reassuring fetal testing [10].

RETRACTED

Informed written consent was obtained from each participant. Eligible women were randomized to either: the group taking Azithromycin 1000 mg PO once followed by placebo PO daily for four days (Group I) or that taking Azithromycin 500 mg PO once, followed by Azithromycin 250 mg PO daily for four days (Group II)**.** Randomization was conducted using a computer-generated table of random numbers. Allocation was concealed using closed sealed envelopes that the senior researcher opened after patients' recruitment. Blinding of the participant was done. Both groups received medications for equal durations. The Azithromycin and placebo (containing starch) were prepared in capsule form with a similar appearance, taste, size, and color. They were prepared in strips and numbered according to the list generated by the computer system. Each participant was assigned an order number and received the treatment with the same number.

Eligible women had their detailed history taken and underwent systemic examinations, including general and abdominal examinations. Then, the participants underwent ultrasonography to assess fetal biometry, amniotic fluid volume, and biophysical profiles and exclude any gross fetal anomalies. As baseline investigations, complete blood counts, urine analysis, and C-reactive protein measurements were performed.

Two hundred and ten (210) women were divided randomly into two equal groups, with both groups receiving ampicillin 2 g IV every 6 h for two days (Unasyn 1.5 g, Pfizer, Egypt). The participant in group I received Azithromycin 1000 mg PO once (Xithrone 500 mg, Amoun, Egypt), and those in Group II received Azithromycin 500 mg PO once, followed by azithromycin 250 mg PO daily for four days (Xithrone 500 mg, Amoun, Egypt).

RETRACTED

The participants were admitted to our hospital. We followed up on the cases to detect maternal and fetal complications (preclinical chorioamnionitis or fetal compromise). Maternal pulse and temperature charts, serial CRP measurements twice weekly, CBC twice weekly, the detection of labor pains, and the detection of vaginal bleeding suggesting placental separation were monitored. The presence of established labor, moderate-to-severe bleeding, fetal distress, or intrauterine infection indicated termination of pregnancy.

The primary outcome was the length of the latency period from the diagnosis of PPROM to delivery (days), and the secondary outcomes were the delivery mode, rate of chorioamnionitis, rate of neonatal intensive care unit (NICU) admission, length of stay in the NICU (LOS), number of stillbirths, number of babies with respiratory distress syndrome (RDS) [The presence of clinical (tachypnea, grunting, and cyanosis in the first day of life, required mechanical ventilation including oxygen, continuous positive airway pressure, and mechanical ventilation) and radiological (ground glass opacification, increasing hypo- aeriation, and air bronchograms) signs confirmed the diagnosis of RDS] [11], number of neonatal deaths, and the rate of postpartum endometritis.

The sample size was calculated according to the following formula: [12])

$$\begin{array}{c}n=\frac{\left(\sigma \begin{array}{c}2\\ 1\end{array}+\sigma \begin{array}{c}2\\ 2\end{array}\right){\left(z\frac{a}{2}+z\beta \right)}^{2}}{{\left(\mathrm{log}\left({m}_{1}\right)-\mathrm{log}\left({m}_{2}\right)\right)}^{2}}\\ n=\frac{{\left[\mathrm{log}\left(\frac{1}{2}+\sqrt{\frac{1}{4}+\frac{{\varnothing }_{1}^{2}}{{m}_{1}^{2}}}\right)+\mathrm{log}\left(\frac{1}{2}+\sqrt{\frac{1}{4}+\frac{{\varnothing }_{2}^{2}}{{m}_{2}^{2}}}\right)\right]\left(z\frac{a}{2}{z}_{\beta }\right)}^{2}}{{\left(\mathrm{log}\left({m}_{1}\right)-\mathrm{log}\left({m}_{2}\right)\right)}^{2}}\end{array}$$

**Z α** = 1.96 (The critical value that divides the central 95% of the Z distribution from the 5% in the tail).

**Zβ** = 0.84 (The critical value that separates the lower 20% of the Z distribution from the upper 80%).

**m1**: median number of days of Group 1 receiving Azithromycin 1000 mg single dose (m1 = 4.9) [13].

**m2**: median number of days of Group 2, receiving Azithromycin 500 mg PO once, followed by Azithromycin 250 mg PO daily for four days (m2 = 5) [13].

***σ*2**: the variance of the log-transformed primary outcome for the group.

**φ2**: The variance of the untransformed outcome for the group.

RETRACTED

So, the sample size was 210 cases divided into two equal groups.

## Statistical analysis

The collected data were coded, processed, and analyzed using SPSS (Statistical Package for Social Sciences) version 22 for Windows® (IBM SPSS Inc., Chicago, IL, USA). Data were tested for normality of distribution using the Shapiro–Wilk test. Qualitative data were represented as frequencies and percentages. The chi-square (χ2) test was used to calculate differences between two or more groups of qualitative variables. Quantitative data were expressed as the mean ± SD (Standard deviation). The independent samples t-test was used to compare two independent groups of normally distributed variables (parametric data). Comparisons between quantitative variables were performed using the one-way analysis of variance to test the difference between the means of several subgroups of a variable. *P*-values of < 0.05 were considered statistically significant.

## Results

Initially, there were 234 potential participants; however, 24 of the women did not meet the selection criteria (seven women had multiple pregnancies, four had lethal fetal anomalies, and 13 declined to participate). Two hundred and ten women consented to participate and were divided into two groups. Group I included 105 women, and Group II included 105 women. All participants completed their follow-up visits till the end of the study (Fig. 1).

**Fig. 1:** Patients' flow chart

There was no significant difference in baseline socio-demographic characteristics and obstetric data between the two groups. (Tables 1 and 2).

**Table 1:** Personal data of the participants in the study groups

	**Group I** **(*n* = 105)**	**Group II** **(*n* = 105)**	***P* value**
**Age** (years)			
Mean ± SD	28.61 ± 5.33	28.86 ± 5.51	0.741
Range	19.0–42.0	18.0–43.0	
**Residence**, n (%)			
Urban	28 (26.7%)	20 (19.0%)	0.189
Rural	77 (73.3%)	85 (81.0%)	
**Educational level**, n (%)			
Illiterate	26 (24.8%)	29 (27.6%)	
Basic education	54(51.4%)	53(50.5%)	0.880
Secondary or more	25 (23.8%)	23(21.9%)	
**Work**, n (%)			
Working	23 (21.9%)	21 (20.0%)	0.735
Not working	82 (78.1%)	84 (80.0%)	
**BMI(Kg/m**^**2**^**)**			
Mean ± SD	33.39 ± 4.21	32.84 ± 4.21	0.350
Range	25.3–40.6	25.3–40.6	

*BMI* Body mass index, *kg/m*^*2*^ Kilogram per square meter, *n (%)* Number and percentage, *SD* Standard deviation

**Table 2:** Obstetric data of women in our RCT

Obstetric data	Group I (*n* = 105)	Group II (*n* = 105)	*P*-value
**Parity**			
Mean ± SD	1.70 ± 1.70	1.64 ± 1.59	0.847
Median (Range)	1.0 (0.0–8.0)	1.0 (0.0–6.0)	
**No. of NVD**			
Mean ± SD	1.01 ± 1.47	0.81 ± 1.47	0.253
Median (Range)	0.0 (0.0–6.0)	0.0 (0.0–6.0)	
**No. of CS**			
Mean ± SD	0.70 ± 1.15	0.85 ± 1.22	0.404
Median (Range)	0.0 (0.0–5.0)	0.0 (0.0–5.0)	
**History of CS**, n (%)			
Yes	37 (35.2%)	40 (38.1%)	0.667
No	68 (64.8%)	65 (61.9%)	
**No. of living children**			
Mean ± SD	1.62 ± 1.49	1.57 ± 1.48	0.825
Median (Range)	1.0 (0.0–5.0)	1.0 (0.0–6.0)	
**History of abortion**, n (%)			
Yes	36 (34.3%)	38 (36.2%)	0.773
No	69 (65.7%)	67 (63.8%)	
**Duration from last delivery** (months)			
Mean ± SD	24.72 ± 3.43	23.95 ± 3.50	0.175
Range	18.0–30.0	18.0–29.0	
**Gestational age** (weeks)			
Mean ± SD	32.49 ± 2.96	31.95 ± 3.74	0.252
Range	25.0–36.9	24.3–36.9	
**Gestational age groups:**			
24–28^+6^ wks	10 (9.5%)	22 (21%)	
29–32^+6^ wks	12 (11.4%)	31 (29.5%)	0.0001
33–36^+6^ wks	83 (79%)	52 (49.5%)	

*CS* Caesarian section, *NVD* Normal vaginal delivery, *n (%)* Number and percentage, *SD* Standard deviation

More than 35% of women had vaginitis, and 45% had UTIs. Moreover, 21.5% of them had a history of PROM during previous pregnancies. Collectively, no statistically significant differences were found between the two groups in the rates of vaginitis, UTI, and PROM (Table 3).

RETRACTED

**Table 3:** History of the vaginitis, UTI, and PROM in women who participated in the RCT

Past history	Group I (*n* = 105)		Group II (*n* = 105)		*P*-value
	**No**	**%**	**No**	**%**	
**History of vaginitis in current pregnancy**					
Yes	40	38.1%	38	36.2%	0.775
No	65	61.9%	67	63.8%	
**History of UTI in current pregnancy**					
Yes	48	45.7%	45	42.9%	0.677
No	57	54.3%	60	57.1%	
**History of PROM in previous pregnancy**					
Yes	23	21.9%	20	19.0%	0.608
No	82	78.1%	85	81.0%	

Group I's mean latency period (5.80 ± 5.44 days) was significantly higher than group II's (2.88 ± 2.37, *p* = 0.000). Again, the mean gestational age at the time of delivery was higher in Group I than in group II (35.12 ± 2.86 vs. 32.61 ± 3.86; *p* = 0.000, respectively). The rate of postpartum endometritis was significantly higher in Group II (*p* = 0.003). However, no statistically significant differences were found between the two groups in the rate of chorioamnionitis (*p* = 0.347) and the mode of delivery (*p* = 0.155) (Table 4).

**Table 4:** Maternal outcomes

Maternal outcomes	Group I (*n* = 105)	Group II (*n* = 105)	*P*-value
**Latency period** (days)			
Mean ± SD	5.80 ± 5.44	2.88 ± 2.37	0.0001*
Median (Range)	4.0 (1.8–29.0)	2.5 (1.5–19.0)	
**Chorioamnionitis**, n (%)			
Yes	8 (7.6%)	12 (11.4%)	0.347
No	97 (92.4%)	93 (88.6%)	
**Mode of delivery**, n (%)			
NVD	35 (33.3%)	45 (42.9%)	0.155
CS	70 (66.7%)	60 (57.1%)	
**Gestational age at time of delivery** (weeks)			
Mean ± SD	35.12 ± 2.86	32.61 ± 3.86	0.0001*
Range	25.0–37.0	25.0–37.0	
**Gestational age groups:**			
24–28^+6^ wks	5 (4.8%)	11 (10.4%)	0.001
29–32^+6^ wks	12 (11.4%)	30 (28.6%)	
33–36^+6^ wks	88 (83.8%)	64 (61%)	
**Postpartum endometritis**, n (%)			
Yes	3 (2.9%)	15 (14.3%)	0.003*
No	102 (97.1%)	90 (85.7%)	

^*^ Statistically significant difference (P < 0.05)

*CS* Caesarian section, *NVD* Normal vaginal delivery, *n (%)* Number and percentage, *SD* Standard deviation

CS rate did not differ between both groups (70/105, 66.7% for group I vs 60/105, 57.1% for the other group), *p* value 0.155. Indications for CS for groups I and II were elective repeat CS (52.8% and 66.7%, respectively), fetal malpresentation (8.5% and 3.3%, respectively), cephalopelvic disproportion (5.7% and 1.7%, respectively), fetal distress (5.7% and 11.7% respectively), and failed induction of labor (27.1% and 16.7%, respectively) (*p* value 0.147).

RETRACTED

Table 5 shows the neonatal outcomes of the study. Group I's mean birth weight was significantly higher than in Group II (2476.71 ± 650.76 m vs. 1918.21 ± 773.55; *p* = 0.000). Moreover, group I had a better Apgar score at 5 min than Group II (*p* = 0.000). The rate of NICU admission and length of stay at the NICU were lower in Group I than in Group II (*p* = 0.000, 0.001; respectively). The rate of RDS was significantly higher in group II than in Group I (*p* = 0.000), and better neonatal survival was observed in group I than in group II (*p* = 0.041)**.**

**Table 5:** Neonatal outcome

	**Group I** **(*n* = 105)**	**Group II** **(*n* = 105)**	***P*-value**
**Birth weight** (grams)			
Mean ± SD	2476.71 ± 650.76	1918.21 ± 773.55	0.000*
Range	600.0–3100.0	600.0–3050.0	
**APGAR score at 5 min**, n (%)			
< 7	36 (34.3%)	76 (72.4%)	0.000*
Median	3	3	
≥ 7	69 (65.7%)	29 (27.6%)	
Median	9	8.5	
**NICU**, n (%)			
Yes	27 (25.7%)	58 (55.2%)	0.000*
No	78 (74.3%)	47 (44.8%)	
**Length of stay in the NICU** (days)			
Mean ± SD	4.67 ± 2.97	7.21 ± 2.84	0.001*
Median (Range)	3.0 (1.0–11.0)	7.0 (1.0–12.0)	
**RDS**, n (%)			
Yes	25 (23.8%)	55 (52.4%)	0.000*
No	80 (76.2%)	50 (47.6%)	
**Neonatal survival**, n (%)			
Alive	96 (91.4%)	84 (80.0%)	
IUFD	6 (5.7%)	10 (9.5%)	0.041*
Neonatal death	3 (2.9%)	11 (10.5%)	

^*^Statistically significant difference (P < 0.05)

*CS* Caesarian section, *IUFD* Intrauterine fetal death, *NICU* Neonatal intensive care unit, *NVD* Normal vaginal delivery, *n (%)* Number and percentage, *RDS *Respiratory distress syndrome, *SD* Standard deviation

## Discussion

The latency period and mean gestational age at delivery were significantly higher in group I than in group II. The rate of postpartum endometritis was higher in group II than in group I. No statistically significant differences in the rate of chorioamnionitis and mode of delivery were noted between the two groups. Better neonatal outcomes were observed in group I than in group II. An earlier study reported a non-significant difference in latency or maternal and neonatal outcomes between women with PPROM at 24–34 weeks of gestation who were given either Azithromycin (*n* = 29) or Erythromycin (*n* = 67) [14]. Pierson et al. reported equivalent outcomes between Azithromycin and Erythromycin, favoring Azithromycin as a substitution for the original seven-day Erythromycin [7]. However; the previous two studies were retrospective that compared two different drugs in PPROM (Azithromycin vs. Erythromycin), while the current one compared two dosing regimens of Azithromycin in the management of PROM. It supported our study in the reliance on Azithromycin as a powerful and effective alternative in managing PPROM.

RETRACTED

Another study reported similar latency period among patients with PPROM using Azithromycin or Erythromycin. The only differences were in maternal and neonatal outcomes being the higher cesarean delivery rates and positive neonatal blood cultures in the erythromycin group [8]. Also, this study was a retrospective cohort one comparing two different drugs in the management of PPROM. However, they used Azithromycin in a dosing regimen similar to ours in the one-day Azithromycin group. Comparisons of the results of the azithromycin group of this study with those of our one-day azithromycin group revealed that the range of the latency period in our study was 1.8–29 days vs. 3.1–12.1 days. We had a higher rate of CS deliveries (66.7% vs. 29.5%), lower rate of chorioamnionitis (7.6% vs. 24.2%), lower rate of neonatal RDS (23.8% vs. 64.5%), and a lower rate of neonatal death (2.9% vs. 4%) [8].

An earlier multicenter, retrospective cohort study compared different dosing regimens of Azithromycin (single dose, 5 day regimen, and 7 day regimen) with Erythromycin in the management of PPROM. They demonstrated no significant difference in either latency to delivery, gestational age at the time of delivery, or the incidence of chorioamnionitis. According to neonatal outcomes, RDS was more common in the five-day azithromycin group. The five-day azithromycin group showed a lower proportion of neonates with five-minute Apgar scores of < 7 and a shorter length of stay in the NICU compared with other groups [13]. Regarding neonatal outcomes, in line with our findings, RDS was more common in the five-day azithromycin group. However, in contrast to our results, the five-day azithromycin group showed a lower proportion of neonates with five-minute Apgar scores of < 7 and a shorter length of stay in the NICU compared with other groups. Although neonatal outcomes were improved in group I, other factors would be implicated as the gestational age at rupture of membranes, latency period, and fetal weight [15].

RETRACTED

In addition, azithromycin was associated with a decreased risk for developing clinical chorioamnionitis, neonatal sepsis, and postpartum endometritis with no difference in the latency period compared with erythromycin. However; these studies combined these antibiotics with ampicillin and amoxicillin [16–18]. There was no difference between the current study and these ones regarding the latency period but maternal and neonatal outcomes varied. This would be rendered to the combined use of ampicillin and amoxicillin with Azithromycin while the current study used Azithromycin alone. Additionally, the intravenous rout for azithromycin even when combined with ampicillin, would explain the variability in the maternal and neonatal outcomes between both studies [18].

The gestational age at PROM was inversely related to the latency period [19]. Despite rupture of membranes at advanced gestational age was reported predominantly in group I (79%), the latency period was significantly prolonged in this group. This would be rendered to the effect of Azithromycin therapy as evidenced previously [20] besides, an earlier study failed to report a correlation between the latency period and the gestational age at rupture of membranes [21].

Azithromycin has some properties that make it superior for treatment of PROM. It has a wide proper antimicrobial coverage that has been described as similar to erythromycin, the first line drug for the treatment of PROM. Also, it has a longer half- life (3 days) especially in the myometrium (70 h). In addition, it has better tolerability due to decreased gastrointestinal side effects [22, 23]. This contributes to the effectiveness of azithromycin especially for the high single dose which is associated with high tissue concentrations and persistent therapeutic levels for longer durations [24]. However; there is no standard regimen for Azithromycin therapy leading to variable dosing regimens [13] which mandates further studies to define the proper dosing regimen.

## Strengths and limitations

Our study is the first registered clinical trial focused on the effect of the use of two different regimens of Azithromycin with a large number of patients (210) over 17 months. Better results could be obtained if future clinical trials, including more cases and of a multicentric nature, are carried out to compare different dosing regimens of Azithromycin in the expectant management of PPROM. Long term neonatal follow up was lacking.

## Research implications

Further multi-center studies with a larger number of patients would be recommended to determine the promising effect of single-dose Azithromycin in managing PPROM.

RETRACTED

## Conclusions

Azithromycin given in a single initial dose, effectively prolonged the latency period, decreased the incidence of chorioamnionitis in women with PPROM at 24–36 + 6 weeks of gestation.

## Data Availability

The datasets generated and/or analyzed during the current study are included in this published article and available in attached supplementary file.

## Abbreviations

PO: Per oral
RDS: Respiratory distress syndrome
PPROM: Preterm premature rupture of membrane
ROM: Rupture of membranes
IGFBP-1: Insulin-like growth factor-binding protein-1
PAMG-1: Placental alpha microglobulin-1
ACOG: American College of Obstetricians and Gynecologists
CRP: C- reactive protein
CBC: Complete blood count
NICU: Neonatal intensive care unit
LOS: Length of stay in the NICU
PROM: Premature rupture of membrane
CS: Cesarean delivery

## References

[1] ACOG Committee on Practice Bulletins-Obstetrics. ACOG Practice Bulletin No. 80. premature rupture of membranes. Clinical management guidelines for obstetrician-gynecologists. Obstet Gynecol. 2007;109:1007–19.17400872 10.1097/01.AOG.0000263888.69178.1f

[2] Mercer BM. Preterm premature rupture of the membranes. Obstet Gynecol. 2003;101:178–93.12517665 10.1016/s0029-7844(02)02366-9

[3] Thomson AJ. On behalf of the Royal College of Obstetricians and Gynaecologists. Care of women presenting with suspected preterm prelabour rupture of membranes from 24+0 weeks of gestation. BJOG. 2019;126:e152–66.31207667 10.1111/1471-0528.15803

[4] National Institute for Health and Care Excellence. Preterm labour and birth NG25; 2015. www.nice.org.uk/guidance/ng25. Accessed 15 May 2017.26632624

[5] Kenyon SL, Boulvain M, Neilson J. Antibiotic treatment in premature rupture of membranes: a systematic review. Obstet Gynecol. 2004;104:1051–7.15516401 10.1097/01.AOG.0000143268.36682.21

[6] Mercer BM. Preterm premature rupture of the membranes: current approaches to evaluation and management. Obstet Gynecol Clin North Am. 2005;32:411–28.16125041 10.1016/j.ogc.2005.03.003

[7] Pierson RC, Gordon SS, Haas DM. Retrospective comparison of antibiotic regimens for preterm premature rupture of membranes. Obstet Gynecol. 2014;124:515–9.25162251 10.1097/AOG.0000000000000426PMC4147675

[8] Finneran MM, Appiagyei A, Templin M, Mertz H. Comparison of Azithromycin versus Erythromycin for prolongation of latency in pregnancies complicated by preterm premature rupture of membranes. Am J Perinatol. 2017;34:1102–7.28637060 10.1055/s-0037-1603915

[9] Romero R, Chaemsaithong P, Korzeniewski SJ, Kusanovic JP, Docheva N, Martinez-Varea A, Ahmed AI, Yoon BH, Hassan SS, Chaiworapongsa T, Yeo L. Clinical chorioamnionitis at term III: how well do clinical criteria perform in the identification of proven intra-amniotic infection? J Perinat Med. 2016;44(1):23–32. 10.1515/jpm-2015-0044.PMID:25918914;PMCID:PMC5881919.25918914 10.1515/jpm-2015-0044PMC5881919

RETRACTED

[10] Bond DM, Middleton P, Levett KM, et al. Planned early birth versus expectant management for women with preterm prelabour rupture of membranes prior to 37 weeks gestation for improving pregnancy outcome. Cochrane Database of Syst Rev. 2017;17:CD004735.10.1002/14651858.CD004735.pub4PMC646469228257562

[11] Sweet D, Bevilacqua G, Carnielli V, Greisen G, Plavka R, Saugstad OD, et al. European consensus guidelines on the management of neonatal respiratory distress syndrome. J Perinat Med. 2017;35(3):175–86.10.1515/JPM.2007.04817480144

[12] - Aidan G. O'Keeffe, Gareth Ambler and Julie A. Barber (2017): Sample size calculations based on a difference in medians positively skewed outcomes in health care studies. O'Keeffe et al. BMC Medical Research Methodology (2017) 17:157. DOI 10.1186/s12874-017-0426-110.1186/s12874-017-0426-1PMC571217729197347

[13] Navathe R, Schoen CN, Heidari P, et al. Azithromycin vs Erythromycin for the management of preterm premature rupture of membranes. Am J Obstet Gynecol. 2019;221:1–8.30904320 10.1016/j.ajog.2019.03.009

[14] Gelber S, Brent E, Varrey A, Fridman B, Sapra K, Frayer W. Equivalence of Erythromycin and Azithromycin for treatment of PPROM. Am J Obstet Gynecol. 2013;208:291.

[15] Esteves JS, de Sá RA, de Carvalho PR, Coca Velarde LG. Neonatal outcome in women with preterm premature rupture of membranes (PPROM) between 18 and 26 weeks. J Matern Fetal Neonatal Med. 2016;29(7):1108–12.26138545 10.3109/14767058.2015.1035643

[16] Martingano D, Singh S, Mitrofanova A. Azithromycin in the treatment of preterm prelabor rupture of membranes demonstrates a lower risk of chorioamnionitis and postpartum endometritis with an equivalent latency period compared with erythromycin antibiotic regimens. Infect Dis Obstet Gynecol. 2020;2020:2093530.32694907 10.1155/2020/2093530PMC7368187

[17] Sinrat N. The outcomes of ampicillin plus Azithromycin to prolong latency period in preterm premature rupture of membranes between 24 and 33+6 weeks of gestation at King Chulalongkorn Memorial Hospital. Thai J Obstet Gynaecol. 2020;28:175–82.

[18] Kole-White MB, Nelson LA, Lord M, et al. Pregnancy latency after preterm premature rupture of membranes: oral versus intravenous antibiotics. Am J Obstet Gynecol MFM. 2021;3(3):100333. 10.1016/j.ajogmf.2021.100333.10.1016/j.ajogmf.2021.10033333607320

[19] Davis JM, Krew MA, Gill P, Nelson KM, Hopkins MP. The role of continuous fetal monitoring in the management of preterm premature rupture of membranes. J Matern Fetal Neonatal Med. 2008;21:301–4.18446655 10.1080/14767050802022789

RETRACTED

[20] Atarjavdan L, Khazaeipour Z, Shahbazi F. Correlation of myometrial thickness and the latency interval of women with preterm premature rupture of the membranes. Arch Gynecol Obstet. 2011;284:1339–43.21298281 10.1007/s00404-011-1841-x

[21] Phupong V, Kulmala L. Factors associated with latency period in preterm prelabor rupture of membranes. J Matern Fetal Neonatal Med. 2016;29(16):2650–3.26482892 10.3109/14767058.2015.1095884

[22] Vogel JP, Nardin JM, Dowswell T, West HM, Oladapo OT. Combination of tocolytic agents for inhibiting preterm labour. Cochrane Database Syst Rev. 2014;(7):CD006169. 10.1002/14651858.CD006169.pub2.10.1002/14651858.CD006169.pub2PMC1065748425010869

[23] - Labs P. Zithromax (R) highlights of prescribing information. 2013. Available at: https://www.accessdata.fda.gov/drugsatfda_docs/label/2013/050710s039,050711s036,050784s023lbl.pdf. Accessed Sept. 17, 2018.

[24] Schreiber H, et al. Macrolide antibiotics roxithromycin vs. azithromycin for preterm premature rupture of membranes: a retrospective comparison. Arch Gynecol Obstet. 2019;300(3):569–73. 10.1007/s00404-019-05221-w.31227871 10.1007/s00404-019-05221-w

